# Honey on Basketball Players' Physical Recovery and Nutritional Supplement

**DOI:** 10.1155/2022/6953568

**Published:** 2022-02-10

**Authors:** Huaming Tang

**Affiliations:** College of Physical Education, Southwest University, Beibei 400715, Chongqing, China

## Abstract

Sports injury is a subject that every athlete will face, and it is the easiest to happen in training and competition, especially for basketball players. Moreover, the excessive fatigue caused by sports not only reduces the person's ability to play sports, but also it reduces the person's participation in normal training and competition. Sugar and fat play a dominant role in energy metabolism, while protein only plays an auxiliary role. For competitive sports, sugar is the most important energy, and the main components of honey are glucose and fructose. Therefore, this paper attempts to explore the effect of honey on the physical recovery and nutritional supplement of basketball players. In this paper, 10 basketball players in our city were selected as the experimental objects and the data of their physiological and biochemical indexes were analyzed. The results showed that the average hemoglobin of the experimental group decreased from 14.45 g·100 ml^−1^ in the first week to 13.23 g·100 ml^−1^ in the second week, increased to 14.25·100 ml^−1^ in the third week, and increased to 15.79.100 ml^−1^ in the fourth week. Adding honey can improve the content of HB and CK of basketball players in higher vocational colleges and reduce the increase of BUN, to slow down fatigue and accelerate the speed of physical recovery.

## 1. Introduction

In the basketball match, the rhythm of the match is accelerated, the antagonism of the players is enhanced, and the competition in time and space is bound to be more intense. Only when athletes have a high level of physical development can they adapt to the needs of modern basketball competition. The low level of physical fitness is a common problem of basketball players in China. There is still a big gap between the level of physical fitness of Chinese athletes and the world-class level. There are still many deficiencies in physical training, especially the lack of scientific and effective systems for athletes' physical recovery and nutrition supplements.

There is no training without recovery. Increasingly, coaches have gradually realized the importance of delaying athletes' fatigue and promoting their physical recovery through nutrition and other measures [1]. Shaw discusses the impact of the Australian Sports Association's sport supplement program on the supplementary exercise of Australian elite swimmers and compares it with other athletes of the same national team [2]. The results show that this supplementary item has played a certain role in swimmers and other athletes, mainly in supplementing nutrition. Karoff et al. surveyed 100 low-income Spanish speaking people living in the United States who have a low level of English, mainly of Mexican origin. Participants reported on their nutrition and exercise self-efficacy, Spanish health literacy, nutrition, and physical activity behavior [3]. Their research shows that participants still pay more attention to physical nutrition supplements. The self-efficacy of exercise means that people will maintain exercise if they attribute the improvement of their physical condition to their active exercise. The comprehensive health program at the University of Miami's Sylvester Comprehensive Cancer Center aims to provide comprehensive health education to cancer patients, survivors, and caregivers by providing guidance on exercise, nutrition, and complementary and alternative medicine. Stoutenberg aims to assess the impact of IWP on the overall health of individuals participating in the program. Stoutenberg's research shows significant improvements related to eating habits. Combined with the results of the participants' satisfaction surveys, IWP has been widely recognized and can positively affect the overall health of cancer patients, survivors, and their caregivers [4]. The purpose of this study is to point out that nutritional supplements may be a more healthy, sustained, and effective method to improve the physical condition. In this article, there is some theoretical support to prove the effect of nutritional supplements on human body. Witard and Ball discusses plant-based protein sources to offset age-related muscle mass loss, and the links between nutrition, exercise, and brain function, illustrating the link between nutrition/exercise and insulin resistance and human models. Finally, Witard and Ball explored the combined effects of nutrition and exercise on reducing the risk of type 2 diabetes and dyslipidemia. On the whole, the interaction between diet and physical activity is more beneficial to human health than simple physical activity [5]. The final result of this study shows that maintaining human health needs the interaction of nutrition supplements and exercise. All above studies are aimed at “the role of nutritional supplements in maintaining human health balance”, and their research methods and results provide important methodological guidance and theoretical support for this paper.

Honey is a supersaturated solution of sugar, which will produce crystallization at low temperature. The part of crystallization is glucose, and the part without crystallization is mainly fructose [6]. Honey has been used medicinally for thousands of years. The beneficial effects of honey, especially its antibacterial activity, indicate that it is a useful choice for the treatment of various wounds. This paper reviews the mechanism and therapeutic effect of honey in wound healing. Laboratory studies and clinical trials have shown that honey can promote autolysis debridement, stimulate wound tissue growth, and stimulate anti-inflammatory activity, thus accelerating the wound healing process. Honey is more effective in eliminating microbial contamination, reducing wound area, and promoting re-epithelization compared with external preparations such as hydrogen fiber, silver, or silver sulfadiazine. In addition, honey improves wound healing by reducing the incidence rate and excessive scar formation. Therefore, the application of honey is an economical and effective method for the treatment of large and complex wounds [7]. Gulfraz et al. collected 40 samples of different types of honey from different parts of Pakistan. The composition of honey samples also changed due to different flora [8]. Deng et al. have established a new platform for direct and rapid detection of tetracycline in honey samples by neutral desorption extraction electrospray ionization mass spectrometry [9]. Orso et al. developed a simple, rapid, and efficient method for the simultaneous determination of 13 antibiotics in honey samples. The method has been successfully applied to real samples from different plants and geographical sources, and combined with the advantages of selectivity and sensitivity of uhplc-ms/MS, it is suitable for routine analysis [10].

Because the main components of honey are glucose and fructose, it will be the focus of this paper to turn it into a nutritional preparation for supplementing sugar during basketball matches and training. Based on the comparison of the physiological and biochemical indexes between the experimental group and the control group, this paper obtains the effective data of the physical reaction of basketball players taking honey, to seek a more scientific and reasonable theoretical basis for honey as a nutritional supplement in basketball.

## 2. Basketball Player Honey

### 2.1. Physical Fitness of Basketball Players

Basketball was invented by American James Naismith in 1891. At that time, he taught at the YMCA International Training School in Springfield, Massachusetts. Because the local area is rich in peaches, the children here like to play the game of throwing balls into the peach basket very much. This inspired him and learned from the characteristics of other ball games such as football and hockey, and created basketball games. The basketball match time is long, the field is small, and the offensive and defensive confrontation is fierce, which requires the aerobic function of athletes. At the same time, at the moment when most basketball technical movements are completed, such as breakthrough, it is the extreme intensity exercise, which is the anaerobic energy supply of ATP-CP and glycolysis system. Athletes need to have good anaerobic energy supply and lactic acid energy recovery ability. The characteristics of basketball determine that the physical quality of athletes is very high. Good endurance level is the basis of long-term repeated high-intensity sports; strength is the guarantee of confrontation ability; speed plays an important role in the improvement and improvement of competitive ability; agility is conducive to stress response and emergency handling on the basketball court; and flexibility can help athletes better adapt to the heavy load and strong confrontation competition. Play a buffer role, and reduce the generation of damage [11].

Basketball players' physical training generally includes physical quality training and special physical quality training, and according to the competition requirements, offensive position, and characteristics, it needs muscle training, speed training, bouncing training, endurance training, etc. Specifically, positioning bench press and squat extreme strength training will be conducted.

Most of the coaches and players do not pay enough attention to physical training. Some coaches have a vague understanding of physical training, and the training plan is not perfect enough to consider the growth and development characteristics of teenagers. The coaches in our country do not pay enough attention to the physical training of basketball. The performance of coaches in the team configuration is not reasonable, tactical training instead of physical training, and the theoretical knowledge of basketball is not comprehensive enough [12].

Body work can cause adaptation changes in many organ systems in the body. The adaptability of these systems not only reflects the ability of body work, but also reflects the physical state of athletes. The adaptive changes of skeletal muscle tissue, cardiovascular system, and respiratory system occur when the body does work, which makes the blood content of muscle increase with the load of material metabolism. The increase of blood flow does not occur immediately at the beginning of exercise, and most of it needs a certain starting time. At the end of the start-up phase, the blood flow can approximately meet the demand during low load exercise. In the high load exercise, the demand cannot be met, and the insufficient blood flow will cause the change of muscle material metabolism. In low load physical exercise, after the start time of anaerobic system function, there is an energy supply of the aerobic system. At this time, muscle not only uses glucose, but also fatty acids and glycerol. In high load physical exercise, a considerable part of energy is obtained by anaerobic system metabolism. The energy supply of anaerobic system can cause muscle blood flow insufficiency, blood oxygen saturation decrease or aerobic metabolism narrow path, lactic acid production increase causes muscle fatigue, and then causes exercise fatigue.

The normal metabolism and good nutritional status of the body are the important for maintaining life activities. In competitive sports, the metabolism of the body is extremely vigorous, which shows that sports nutrition is different from the general public nutrition on the basis of basic nutrition, that is, there are higher requirements for nutrition demands and supplements. Any metabolic disorder or malnutrition can affect the function of tissue cells. The nutritional status of the body is closely related to the athletic state of athletes. Nutritional supplements should not only improve physical fitness in the process of training, but also be beneficial to sports recovery. Moreover, when the body's nutritional needs cannot maintain the body's metabolism and growth and development needs, it is necessary to take in enough calories and various nutrients through additional ways or supplement special nutritional preparations to meet the needs of maintaining the function, structure, metabolism, and movement of body cells. Athletes' physical fitness is affected by training, heredity, nutrition, and other factors. Scientific training and nutritional support are two important factors to improve the physical fitness of basketball players. One of the most important means to develop and improve physical fitness is through scientific training.

### 2.2. Honey

Honey is a kind of natural product which is produced by the honeybee by fully brewing the juice secreted by plant nectar collected by bees. It contains rich nutrients, including organic acids, flavonoids, and phenolic acids. These phytochemicals have many functional activities beneficial to human health. Amino acids are a kind of small molecular compounds in honey. They are mainly derived from the pollen of flowering plants and are greatly affected by the climate and soil of flower source plants. In addition to protein amino acids, there are some nonprotein amino acids in honey. Protein amino acids include 8 essential amino acids and 12 nonessential amino acids. Nonprotein amino acids are a class of amino acids that do not participate in the formation of proteins. Protein is a kind of trace substance in honey. Its species and content are affected by many factors, such as honey, flower plants, honeybee species, soil, and climate. The protein content is also affected by processing and storage conditions, and amylase is also used as an index to evaluate the freshness of honey. Because of the difference of protein in different honey, protein can be used as a kind of flower source marker of honey, which provides the basis for the identification of flower source and adulteration of honey. Hot processing can induce a variety of reactions, affecting the appearance and flavor of honey. The Maillard reaction between reducing sugar and nitrogenous compounds in honey will occur when heated to form brown substances such as 5-hydroxymethylfurfural. High temperature can accelerate Maillard reaction, so there are a lot of Maillard products in the honey which is over processed, which will affect the color of honey. In addition, the caramel reaction of fructose and the reaction of iron salt and tannate can also affect the color of honey. Hydroxymethyl furfural is a Maillard product under acidic conditions. The pH value of honey is less than 7 and it is acidic. 5-HMF will be generated by Maillard reaction in the process of processing and storage. Therefore, 5-hm is often used as the evaluation index of honey freshness in many standards. 5-HMF is formed by isomerization, double bond breaking, and dehydration of hexose and nitrogen-containing compounds under acidic conditions. The heating temperature and time have a direct effect on the formation rate of 5-HMF. 5-HMF absorbed by the human body will stimulate the skin. At the same time, 5-HMF has neurotoxicity, which can combine with the protein in the human body to cause accumulated poisoning and damage the striated muscle and internal organs of the human body.

Honey is an important secondary metabolite of plants produced by bees. It is composed of more than 100 substances with high nutritional and preventive value. Phenolic compounds are an important class of substances, which help to distinguish people's sensory characteristics. Phenolic compounds can also form some antibacterial and antioxidant substances. At the same time, honey also contains various kinds of organic acids, which play an important role in the control of digestive enzymes and microbial reproduction, so honey is a kind of natural health care product. Because of its sweetness, color, and flavor, honey is also used as a sugar substitute in many manufactured foods. Honey has valuable nourishing, healing, and preventive properties, which are determined by its chemical composition. The content of polyphenols in honey is strongly influenced by the flower and geographical origin as well as the climatic characteristics of the site. Natural honey has a special floral smell, mainly from different volatile small molecular compounds, which belong to different chemical groups. Due to the variety of honey, the newly discovered volatile components are still increasing. It is difficult to distinguish honey from different sources by using a single volatile component, and the concentration of volatile compounds in honey is mostly low, which makes honey complex and difficult to analyze.

This chapter takes 10 elements such as Na, Mg, P, K, Ca, Mn, Zn, Rb, Sr, and Ba as examples, and uses the “bottom-up” method to evaluate the uncertainty of the content of elements in ICP-MS in honey. Honey contains a large number of essential elements of the human body, and the highest content is the K element. K element is one of the important electrolytes in the human body and it takes a major role to maintain the physiological activities of cells. It plays an important role in maintaining the normal osmotic pressure and acid-base balance, maintaining the stability of the internal environment, participating in the metabolism of sugar and proteins, ensuring the normal function of neuromuscular, and so on. Taking the determination of K element in honey as an example, the calculation method of uncertainty is proposed below. First, determine that the K element is determined by

(1) $$\begin{array}{c} \mathrm{w=}\frac{\left(\mathrm{c*}\left(v/m\right)\mathrm{*f}\right)}{R}, \end{array}$$

wherein *w* is the concentration of K elements in honey in mg/kg^−1^, *c* is the concentration of K elements in the solution in mg/L^−1^, *v* is the fixed volume of honey samples in mL, *m* is the quality of honey samples in *g*, *f* is the dilution factor, and *R* is the recovery rate. Three parallel samples were dissolved per honey sample, with Class *A* uncertainties of

(2) $$\begin{array}{c} u\left(A\right)=\frac{\mathrm{SD}}{\sqrt{n}}. \end{array}$$

Relative uncertainty is

(3) $$\begin{array}{c} U\left(A\right)=\;\frac{U\left(A\right)}{w}=\frac{S\;D}{\left(\sqrt{n}*w\right)}=0.79\%. \end{array}$$

According to the balance measurement certificate, the linearity of the balance is ±0.2 mg, calculated according to the uniform distribution, and its uncertainty is

(4) $$\begin{array}{c} u_{1}\left(m\right)=\frac{0.2}{\sqrt{3}}=0.12mg. \end{array}$$

The balance has a resolution of 0.1 mg and is calculated evenly with uncertainties of

(5) $$\begin{array}{c} u_{2}\left(m\right)=\frac{0.1}{\sqrt{3}}=0.058mg\sqrt{a^{2}+b^{2}}. \end{array}$$

The standard uncertainty of the resulting weighing is

(6) $$\begin{array}{c} u\left(m\right)=\sqrt{u_{1}{\left(m\right)}^{2}+u_{2}{\left(m\right)}^{2}}=0.13mg. \end{array}$$

The actual sample size is 1 g, so the relative standard uncertainty of the weighing is

(7) $$\begin{array}{c} U\left(m\right)=\;\frac{U\left(m\right)}{m}=0.012\%. \end{array}$$

Recovery rates (*R*, %) were 94.07, 96.35, 95.96, 96.40, 101.86, and 91.03.

(8) $$\begin{array}{c} B_{+}=R_{\max}-100\%=1.78\%,\\ B_{-}=100\%-R_{\max}=8.46\%,\\ U\left(R\right)=\sqrt{\frac{{\left(B_{+}+B_{-}\right)}^{2}}{12}}=3.42\%. \end{array}$$

*R* is the result of the average recovery rate, which is relatively uncertain:

(9) $$\begin{array}{c} U_{\text{rel}}\left(R\right)=\frac{U\left(R\right)}{\bar{R}}=3.16\%. \end{array}$$

According to the production trademark data, the capacity bottle is marked at 20°C, the capacity tolerance of the Class *A* 50 mL capacity bottle is ±0.05 mL, and since no confidence level or distribution information is given, the uncertainty is assumed to be a triangular distribution:

(10) $$\begin{array}{c} U_{f-50}\left(v\right)=\frac{0.056}{\sqrt{6}}=0.02\text{ ml}. \end{array}$$

The expansion coefficient of water is 2.1 × 10^−4^/C, the capacity bottle is labeled at 20°C, and assuming the laboratory temperature changes to ±4°C, the temperature causes a volume change of 2 ± (50 × 4 × 2.1 × 10-4) and 0.042 mL. Assuming an even distribution, the standard uncertainty of the volume change of the capacity bottle is

(11) $$\begin{array}{c} U_{\text{temp}-50}\left(v\right)=\frac{0.042}{\sqrt{3}}=0.03\text{ ml}. \end{array}$$

Therefore, the uncertainty introduced by the 50 mL capacity bottle fixing capacity is

(12) $$\begin{array}{c} U_{s-50}\left(v\right)=\sqrt{u_{f-50}{\left(v\right)}^{2}+u_{\text{temp}-50}{\left(v\right)}^{2}}=0.029\text{ ml}. \end{array}$$

The relative uncertainty introduced by the 50 mL capacity bottle fixing capacity is

(13) $$\begin{array}{c} U_{\text{rel}-s-50}\left(v\right)=\frac{u_{s-50}\left(v\right)}{v_{s-50}}=0.057\%. \end{array}$$

### 2.3. Physical Recovery and Nutrition Supplement for Basketball Players

As the three major energy supply substances, sugar is an important energy supply material for exercise, while the energy supply of fat to the body appears when the exercise time is prolonged and becomes the main energy supply material. A large amount of sugar energy is consumed at the beginning of exercise, and with the extension of exercise time, the supply of fat to the body capacity increases, but when the final sprint stage is reached, sugar is still the main energy supply. Not only basketball, but also for almost every sport, sugar supplement energy consumption is the first, while fat is the second. Basketball players should take high sugar food as the main ingredient in their daily diet, but they should also pay attention to the excessive involvement of sugar and the need to supplement nutrients comprehensively.

Basketball players for a long time and high intensity of these movements will inevitably cause athletes to produce physical fatigue, thus affecting the quality of technical movements. In this state, a proper sugar supplement can delay the fatigue, accelerate the recovery of physical strength, and make the athletes complete the competition with higher quality. In the game, basketball players need to exercise frequently and run repeatedly, which will make them sweat too much, cause dehydration and electrolyte disorder, and reduce physical strength in a short time, thus affecting the overall performance of the game. Therefore, athletes should be allowed to drink a small amount of water in the interval of competition, to prevent the athletes from dehydration, to ensure the athletes' good competitive state. The best time for sugar supplement is within two hours after the competition. In addition, continuous supplement should be conducted at regular intervals. In addition, the amount of sugar should be supplemented according to the weight of different individuals. This kind of sugar supplement after the competition, which consumes a lot of physical fitness, is conducive to the rapid recovery of physical fitness, and is also very helpful to the athletes' training and competition in the next stage.

## 3. Experiment Materials and Methods

### 3.1. Subjects

For the selection of experimental subjects, men and women are not included at the same time. Although boys and girls have different body structures, they are the same in terms of nutritional supplements and body composition. This paper selects 10 men's basketball team members of our city's Mass Media Vocational and Technical College as the research object. In order to ensure the reliability of the experimental conclusion, different training years and age stages of basketball majors should be considered when selecting athletes. The average age is between 18 and 22 years, and the training period is two to six years. They were divided into two equal height groups, one group as the experimental group supplemented with honey, the other group as the control group without honey supplement. All athletes volunteered to participate in the test. According to the physical examination report of freshmen, we can confirm that the subjects have no history of cardiovascular system, liver and kidney diseases, and lung disease. During the training period, the diet of athletes is arranged by the coach group, and the diet and daily life of the players are strictly controlled. There was no significant difference in height, weight, age, and training years between the two groups.

### 3.2. Experimental Methods

Ten basketball players were trained for months. They had a rest every Sunday and trained twice a day. The main training was physical fitness training. This paper takes the training cycle of this month as the research period, takes the weekly training plan as the unit, and trains four weeks of the same plan. Each person took 300 ml honey three times a day. The physiological and biochemical indexes were tested before morning training on Monday, while the indexes of physical fitness and strength were measured after the evening training every Saturday. Using the literature, design, survey and interview, and observing the body function, physical fitness, and some physiological and biochemical indexes of the research objects, a comparative analysis was carried out. All data were processed by statistical software, and the standard deviation was calculated. The formula of mean and standard deviation is as follows:

(14) $$\begin{array}{c} \mu =A_{n}=\frac{a_{1}+a_{2}+a_{3}+\cdots +a_{n}}{n},\\ \sigma =\sqrt{\frac{1}{N}\sum_{i=1}^{N}{\left(x_{i}-\mu \right)}^{2}.} \end{array}$$

### 3.3. The Development of Artificial Intelligence to Achieve All-Round Human Development

The development of artificial intelligence and the realization of human freedom and comprehensive development are dialectical unity. The rise of science and technology, represented by artificial intelligence, is conducive to the liberation of mankind, which promotes “the free and all-round development of human beings” by fully manifesting human personality, strengthening human abilities, and broadening the human knowledge horizons. However, the development and progress of artificial intelligence have also led to the “tool rationality” of science and technology instead of human “value rationality,” leading to the existence of the two contradictories. It is necessary to reflect on the problems in the development of artificial intelligence science and technology, determine the reasons for the existence of tool rationality and value rationality phenomenon, and promote people's all-round development. “The free and comprehensive development of human beings” is Marx's profound description of the communist society, and it is also the pursuit of the beautiful social form, reflecting the general course of the society from the lower level to the higher level. The universal phenomenon of people's all-round development becoming a group exists in the same world, and people can freely choose to live in various fields according to their own special skills, so as to realize the value of human's essential abilities.

Based on the above motion capture hardware and software system, this chapter mainly designs the method of human data collection, processing, and application. After the system calibration is complete, different experiments can be designed according to different designs. In the human motion analysis experiment, the marker points should be attached to human skin or special clothing, that is, the appearance of the skin point. The original data collected by the system are the appearance data of the skin. Appearance skin data cannot be directly used for human motion analysis. A feasible method is to estimate the position of human bones, that is, to calculate bone points, and the trajectory of bone points is called bone point data. The bone model analyzes the various movements of the human body and finally optimizes the human motion data for use in humanoid robots, as shown in Figure 1. Motion data capture technology includes contact type and non-contact type, and the basic types include mechanical, electromagnetic, optical, and inertial types.

Software system operation depends on the hardware system to read the human body motion data, and the human body data involved are divided into three categories, namely skin data, joint data, and bone data. Each type of data from bottom to top is divided into three layers, the hierarchy as shown in Figure 2, from bottom to top for the original data, cell data, and overall data. Hierarchical analysis of human body data can be more scientific to analyze the health status of human body from different angles. For example, cell data can find the problems of human body from the micro level. The appearance of the skin point represents the marker point attached to the surface of the human body, and it is different from the original point collected by the system wherein the skin point has the meaning of representing a certain part of the human body, and the original point does not.

The development of artificial intelligence has greatly improved people's ability to transform nature, from the initial physical labor gradually changed to mental labor, the transformation of production mode into human's all-round development has accumulated a large amount of material capital, people's free space is relatively expanded, and people's understanding of the objective world has changed accordingly. The widespread application of artificial intelligence technology for the overall development of human material wealth must not be based on the sacrifice of human subjectivity, and artificial intelligence technology research often reflects the insurmountability of human beings. The emergence of artificial intelligence gives people more time to free up, and use the time saved to do many more meaningful things. It not only improves the efficiency of human work, but also reduces the pressure on people's lives.

## 4. Analysis on the Effect of Honey on the Physical Recovery and Nutritional Supplement of Basketball Players

### 4.1. Dietary Survey and Nutritional Assessment Analysis

Among the five players, only two athletes had proper heat intake, one had a high calorie intake, and the other two had a low calorie intake; only three of the five athletes had a normal carbohydrate intake, and one had a low carbohydrate intake; only three of the five players had a low protein ratio, only two athletes had a high proportion of protein intake; only four of the five athletes had a high proportion of fat intake, and only one athlete's fat intake ratio did not exceed the recommended value. The intake of heat, energy, and three major thermogenic nutrients of basketball players is shown in Table 1.

VB1 can keep the body circulation, digestion, nerves, and muscles normal, constitute the coenzyme of decarboxylase, and participate in sugar metabolism; VB2 is essential for metabolism, energy utilization, and composition of proteins, sugar and fatty acids, and can promote physical development. VPP plays an important role in transferring hydrogen in the process of cell physiological oxidation. VE can maintain normal reproductive capacity and muscle metabolism, and maintain the integrity of the central nervous system and vascular system. There is no obvious problem in athletes' vitamin intake, and the intake of multi-vitamins closely related to sports ability can meet the needs of training days, mainly due to the timely and adequate supplement of corresponding nutrients in the process of training. The analysis of athletes' vitamin intake is shown in Figure 3.

The results of the dietary survey show that the intake of various minerals by athletes can meet the recommended standard. Among them, iron is beneficial to maintain the level of hemoglobin; selenium has an antioxidant effect, which can eliminate the increase of free radicals caused by hypoxia, thus completing the protection of muscle cell membrane. The results show that the calcium, iron, zinc, and selenium of athletes are higher than the recommended value, which is in line with the characteristics that athletes need to increase these minerals when they exercise in a high temperature environment. Some athletes were deficient in calcium and potassium in team 2.

### 4.2. Analysis of Nutritional Recovery of Athletes with Low Immunity

The training with high intensity and large amount of exercise often breaks the balance of the body's original immune function, resulting in immunosuppression, thus reducing the immune function of the body. Exercise has a significant effect on the changes of T cells and B cells. The training with high intensity and large amount of exercise often breaks the balance of the body's original immune function, resulting in immunosuppression, thus reducing the immune function of the body. Exercise has a significant effect on the changes of T cells and B cells. The changing trend of white blood cells of athletes is shown in Figure 4.

Team 4 may have developed chronic fatigue syndrome after long-term training. The reason of chronic fatigue syndrome induced by exercise is not clear, which may be related to the abnormal immune, endocrine, metabolic function, and neuropsychiatric disease. Chronic fatigue syndrome (CFS) is related to some immune diseases, and there are many abnormal humoral immune cell immune indexes. It is found that under the premise of ensuring the athletes' normal training, they have reached a good functional state.

### 4.3. Effect of Honey on Physiological Indexes of Athletes

In this paper, vital capacity, basic heart rate, and blood pressure are selected to characterize the characteristics and laws of the changes in the physical function of basketball players in vocational colleges. The results showed that there were some differences and changes in the scores between the experimental group and the control group. The general trend was that with the increase of training time, the vital capacity was increasing, while the basic heart rate and blood pressure decreased slowly. The effect of honey on Physiological Indexes of athletes is shown in Figure 5.

The results show that there are some differences and changes between the experimental group and the control group, and the lung capacity of basketball players is gradually improved with the training. During the whole training period, the general trend is that the basic heart rate is stable and gradually decreasing, the intensity of the whole training does not exceed the range of the athletes' load, and the athletes' physical functions are good. However, there was no significant difference between the experimental group and the control group in one to two weeks. The control group was higher than the experimental group for three to four weeks. The experimental group athletes' physical recovery and nutritional supplements were better than the control group.

### 4.4. Analysis on the Influence of Honey on Biochemical Indexes of Athletes

For the analysis of biochemical indexes, it should include the changes of vitamin content, protein content, blood sugar, inorganic salts, and other parameters in athletes' bodies. This experiment takes hemoglobin content as the main index to study. The average hemoglobin of basketball players in the experimental group decreased from 14.45 g·100 ml^−1^ in the first week to 13.23 g·100 ml^−1^ in the second week, increased to 14.25·100 ml^−1^ in the third week, and increased to 15.79·100 ml^−1^ in the fourth week. In the control group, the average hemoglobin decreased from 14.74 g·100 ml^−1^ in the first week to 12.91 g·100 ml^−1^ in the second week, increased to 13.92 g·100 ml^−1^ in the third week, and increased by 14.88 g·100 ml^−1^ in the fourth week. The biochemical indexes of basketball players are shown in Table 2. The data around is chosen for analysis because the time around can cover the whole metabolic cycle of the human body, and can more scientifically observe the change process of biochemical indexes in the human body, so it can reflect the regularity.

This paper selects the average value of hemoglobin, blood urea, and creatine kinase to reflect the change characteristics and rules of basketball players' biochemical indexes. The results showed that there were some changes in biochemical indexes between the experimental group and the control group. The analysis of changes of biochemical indexes of basketball players is shown in Figure 6.

The average value of urea nitrogen in the experimental group of basketball players increased from 5.96 mmol L in the first week to 6.23 mmol·L in the second week, 6.44 mmol·L in the third week, and 6.83 mmol·L in the last four weeks, 887 mmol·L, then increased slowly. However, the average value, maximum value, and minimum value of creatine kinase index of athletes are not the same, and the change does not show a certain rule, and the whole change is in a state of fluctuation. The index of the experimental group was a process of slowly rising and then decreasing.

In the experimental group, honey supplementation promoted the active recovery of the body after exercise, prevented the obvious decline of hemoglobin, maintained the normal function of red blood cells, and promoted physical fitness and physical endurance significantly. Compared with the control group, the increase of BUN in the experimental group decreased, which means that the energy supply of sugar in the experimental group was more than that in the control group, and the exercise level of the experimental group was relatively improved. Taking honey can effectively protect muscle fibers from injury, ensure energy supplement during exercise and ATP recovery after exercise, and maintain the balance of energy supply and transfer during and after exercise. Honey supplementation can improve hypoglycemia after exercise, reduce energy consumption, indirectly reduce cell membrane permeability, and then reduce serum CK concentration. According to the actual physical fitness changes of basketball players, after a full nutrition supplement, ten subjects clearly felt that the training state was better.

## 5. Conclusions

Honey supplement can improve the content of Hb and CK, reduce the increase of BUN, improve the function of oxygen transport system, effectively protect muscle fibers from damage, ensure the energy supplement and ATP recovery reaction during and after intense exercise, and keep the balance of energy supply and transfer during and after exercise, to slow down fatigue and accelerate the speed of physical recovery.

Taking honey can stabilize or slow down the basic heart rate of athletes, but has no obvious effect on vital capacity and blood pressure. Honey has no obvious effect on improving the vital capacity and blood pressure of basketball players in higher vocational colleges, which is conducive to stabilizing or reducing the basic heart rate of athletes, promoting fatigue recovery and physical supplements.

If basketball players want to achieve excellent results, energy supply is the basic guarantee, and the energy material mainly comes from diet. Scientific and reasonable diet arrangement plays an important role in improving sports performance and eliminating fatigue as soon as possible. The following points should be paid attention to in a reasonable diet: first, the reasonable intake of nutrients, and the proportion of protein, carbohydrate, and fat in food should be reasonably arranged on the premise of balanced consumption and supply of athletes; the second is to pay attention to the reasonable proportion of heat source, and the ratio of protein, fat, and carbohydrate should be 1 : 1 : 4. The ratio of endurance events should be 1 : 1 : 7, and it must be high in carbohydrate and low in fat. The third is to pay attention to the acid-base balance of food intake. Although this article has carried out the certain research of honey to the basketball athlete's physical fitness recovery and nutrition supplement, how honey helps in the athletes' physical ability the and recovery mechanism needs further research and thorough exploration.

## Figures and Tables

**Figure 1:** A diagram of the human motion data processing process.

**Figure 2:** The hierarchy of human motion data in software.

**Figure 3:** Analysis of athletes' vitamin intake.

**Figure 4:** The changing trend of athletes' white blood cell.

**Figure 5:** Analysis on the influence of honey on athletes' physiological index.

**Figure 6:** Analysis of changes of biochemical indexes of basketball players.

**Table 1:** Basketball players' heat energy and the intake of three heat-generating nutrients.

		Player 1	Player 2	Player 3	Player 4	Player 5
Total calories (kcal/day)	Actual value	3872	2377	1926	3257	3007
	Recommended value	3076	3578	3714	3578	3462
	Actual/recommended (%)	125.88	66.43	51.86	91.03	86.86
Nutrient heating ratio (%)	Protein	11.3	9.2	15.3	11.1	16.2
	Fat	25.7	17.3	42.6	29.4	27.8
	Carbohydrates	62.7	73.4	42.6	58.6	55.3

**Table 2:** Biochemical indicators of basketball players.

Group	Time	HB (g·100 ml^−1^)	BUN (mmol·L)	CK (U·L)
Test group	The first week	14.45 ± 1.47	5.96 ± 0.76	165.62 ± 96.27
Control group		14.74 ± 1.32	5.82 ± 0.24	177.41 ± 67.62
Test group	The second week	13.23 ± 1.15	6.23 ± 1.32	185.36 ± 106.14
Control group		12.91 ± 1.41	6.94 ± 1.62	189.63 ± 126.28
Test group	The third week	14.25 ± 0.81	6.44 ± 1.65	192.33 ± 95.81
Control group		13.92 ± 1.35	7.36 ± 0.94	201.6 ± 146.25
Test group	The fourth week	15.79 ± 0.54	6.83 ± 1.34	163.25 ± 155.71
Control group		14.88 ± 1.52	7.88 ± 1.24	223.54 ± 95.43

## Data Availability

Data sharing is not applicable to this article as no datasets were generated or analyzed during the current study.
